# Early-Life Exposure to Low-Dose Cadmium Accelerates Diethylnitrosamine and Diet-Induced Liver Cancer

**DOI:** 10.1155/2021/1427787

**Published:** 2021-11-28

**Authors:** Hongbo Men, Jamie L. Young, Wenqian Zhou, Haina Zhang, Xiang Wang, Jianxiang Xu, Qian Lin, Yi Tan, Yang Zheng, Lu Cai

**Affiliations:** ^1^Pediatric Research Institute, Department of Pediatrics, University of Louisville School of Medicine, Louisville, KY 40202, USA; ^2^Department of Cardiovascular Disease, First Hospital of Jilin University, Jilin University, Changchun 130021, China; ^3^Department of Pharmacology and Toxicology, University of Louisville School of Medicine, Louisville, KY 40202, USA; ^4^Department of Medicine, University of Louisville School of Medicine, Louisville, KY 40202, USA; ^5^Wendy L. Novak Diabetes Care Center, Louisville, KY, USA; ^6^Department of Radiation Oncology, University of Louisville School of Medicine, Louisville, KY 40202, USA

## Abstract

Maternal exposure to cadmium causes obesity and metabolic changes in the offspring, including nonalcoholic fatty liver disease-like pathology. However, whether maternal cadmium exposure accelerates liver cancer in the offspring is unknown. This study investigated the impact of early-life exposure to cadmium on the incidence and potential mechanisms of hepatocellular carcinoma (HCC) in offspring subjected to postweaning HCC induction. HCC in C57BL/6J mice was induced by diethylnitrosamine (DEN) injection at weaning, followed by a long-term high-fat choline-deficient (HFCD) diet. Before weaning, liver cadmium levels were significantly higher in mice with early-life cadmium exposure than in those without cadmium exposure. However, by 26 and 29 weeks of age, hepatic cadmium fell to control levels, while a significant decrease was observed in copper and iron in the liver. Both male and female cadmium-exposed mice showed increased body weight compared to non-cadmium-treated mice. For females, early-life cadmium exposure also worsened insulin intolerance but did not significantly promote DEN/HFCD diet-induced liver tumors. In contrast, in male mice, early-life cadmium exposure enhanced liver cancer induction by DEN/HFCD with high incidence and larger liver tumors. The liver peritumor tissue of early-life cadmium-exposed mice exhibited greater inflammation and disruption of fatty acid metabolism, accompanied by higher malondialdehyde and lower esterified triglyceride levels compared to mice without cadmium exposure. These findings suggest that early-life exposure to low-dose cadmium accelerates liver cancer development induced by a DEN/HFCD in male mice, probably due to chronic lipotoxicity and inflammation caused by increased uptake but decreased consumption of fatty acids.

## 1. Introduction

Cadmium (Cd) is a nonessential trace metal recognized as one of the top 20 hazardous substances to humans through occupational and environmental exposure. Ingestion is the main source of Cd in individuals without occupational and smoking exposure [1, 2]. Cd damages various organs, with major effects on the kidneys and the liver [3]. The effects of long-term Cd exposure include increased risks of cardiovascular disorders, obesity, diabetes, and cancer [4–8].

In 2020, more than 905,677 new liver cancer cases were registered worldwide, accounting for 4.7% of overall cancer incidence. Globally, liver cancer ranks third in terms of mortality, and among males, it is the second leading cause of cancer death [9]. Hepatocellular carcinoma (HCC) accounts for approximately 75% of all liver cancers [10], and hepatitis virus remains the most important global risk factor for HCC. However, the importance of metabolic risk factors for HCC, including metabolic syndrome, obesity, type 2 diabetes, nonalcoholic fatty liver disease (NAFLD), and environmental exposure to toxic metals, has been gradually appreciated [11].

In previous studies, we exposed adult rats to very low-dose Cd at 20 nmol/kg for 4 weeks and examined the effect on the kidney and liver at the 20^th^, 36^th^, 44^th^, and 52^nd^ weeks postexposure to Cd [12, 13]. Persistent and mild histopathological changes, along with increases in oxidative damage and cell proliferation, were evident at the late stages (40–52 weeks), and these effects were associated with the persistent downregulation of cellular antioxidant systems [12, 13]. In the following study with mice exposed to the same dose of Cd as used for rats, we showed that Cd exposure induced caspase-8 gene promoter hypermethylation and decreased caspase-8 protein expression, leading to decreased hepatic apoptosis and increased preneoplastic lesions. The outcomes were all prevented with methylation inhibitor, 5-aza-2′-deoxyctidene [14]. These findings suggest that chronic exposure to low-dose Cd does not induce remarkable organ or tissue damages, leading to significant lethal effects, but persistently alters cellular functions and signaling pathways, and this observed Cd-altered cellular signaling (i.e., antioxidant and apoptotic pathways) may cause exposed individuals to be more susceptible to stress, disease risk factors (i.e., diet), and disease progression (i.e., carcinogenesis).

In addition to the adverse health effects resulting from an individual directly being exposed to low-dose Cd during adulthood, increasing evidence also indicates that maternal Cd accumulation can affect fetal development and the offspring's health through the placental transfer of Cd and secretion into breast milk [15–17]. For example, offspring of maternal rats exposed to Cd exhibited a compensatory increase in insulin secretion, accompanied by increased circulating nonesterified fatty acids, a sign of insulin resistance, at two months after birth [18]. In another study, Jackson et al. showed that gestational Cd exposure induced weight gain, insulin resistance, and increased circulating triglycerides, similar to what is seen in NAFLD [19].

Considering the chronic increase in cell proliferation found in the liver of Cd-exposed rats and mice, Cd has been classified as a human carcinogen. Whether gestational exposure to Cd disturbs metabolism and leads to the increase in the offspring's susceptibility to cancer induction or development remains unaddressed. Therefore, the present study investigated the impact of early-life exposure to Cd on the offspring's susceptibility to HCC following postweaning HCC induction. To this end, parental C57BL/6J mice were exposed to 5 ppm Cd in drinking water for 16 weeks before pregnancy until weaning. At weaning, the offspring with and without early-life exposure to Cd underwent HCC induction by diethylnitrosamine (DEN) and a high-fat choline-deficient (HFCD) diet. Both male and female offspring in the early-life Cd exposure groups showed body weight gain. The impact of early-life Cd exposure on HCC incidence in male and female offspring was evaluated. Mechanistically, increased fatty acid uptake and decreased fatty acid disposal may accelerate liver cancer.

## 2. Materials and Methods

### 2.1. Animals and Procedures

All animal procedures were approved by the Institutional Animal Care and Use Committee of the University of Louisville, which is certified by the American Association for Accreditation of Laboratory Animal Care. Six-week-old parental male and female C57BL/6J mice were purchased from the Jackson Laboratory (Bar Harbor, ME, USA). Mice were maintained on a 12 h light/dark cycle at controlled temperature conditions. After 1 week, parental male and female mice were divided into two groups: the control group (female = 5, male = 5) and the Cd group (female = 3, male = 3). The mice in the Cd group were exposed to drinking water containing CdCl_2_ (8.15 mg/L for 5 ppm of Cd). After 16 weeks, male and female mice were housed together to mate. At weaning, the control offspring were subdivided into control (female = 10, male = 10) and HCC-induction (Con-Can female = 9, male = 10) groups. Similarly, 9 female and 10 male offspring with early-life Cd exposure (Cd group) were allocated to the HCC induction (Cd-Can) group, as illustrated in Figure 1(a). The Con-Can and Cd-Can group mice received an intraperitoneal injection of DEN at 25 mg/kg immediately after weaning and were fed a HFCD diet (58% kcal from fat), as reported previously [20]. Control offspring received a PBS injection and were fed a normal diet (11.4% kcal from fat). After 23 weeks, three male and three female mice from each group were sacrificed. After 29 weeks, all remaining mice were sacrificed, and their liver and blood were harvested for metal, histopathological, and protein analyses.

### 2.2. Intraperitoneal Glucose Tolerance Test (IPGTT)

Mice were fasted for 6 h, commencing at 8:00 a.m., and then injected intraperitoneally with glucose solution (1 g/kg body weight) for the intraperitoneal glucose tolerance test (IPGTT). After glucose injection, blood glucose levels were monitored at 0 min, 15 min, 30 min, 60 min, 90 min, and 120 min.

### 2.3. Biochemical Analysis of Plasma and Liver Samples

Plasma alanine aminotransferase (ALT), triglyceride, and cholesterol levels as well as hepatic triglyceride levels were measured using commercially available colorimetric kits (Cat#TR71121, Cat#TR22421, Cat#TR13421, Thermo Scientific, Waltham, MA), respectively. Briefly, plasma samples were diluted with the reagents, mixed well, and incubated at 37°C. The absorbance was measured with a microplate reader according to the manufacturer's instructions. Liver samples were extracted with the extract reagent (chloroform : methanol = 2 : 1) at 4°C overnight after being homogenized in 50 mmol/L NaCl (sodium chloride). The samples were vortexed and centrifuged for 20 min the following day, the lower chloroform layer was collected and recorded, and 500 *μ*L of the lower chloroform layer was placed in Eppendorf tubes and evaporated to dryness in the hood. The dried samples were directly dissolved in a triglyceride reagent. The absorbance was then measured with a microplate reader at 500 nm using a 200 *μ*L mix.

### 2.4. Cd Content in Liver Tissues

The Cd content in liver tissues was measured by inductively coupled plasma mass spectrometry (ICP-MS, X Series II, Thermo Fisher, Waltham, MA). All samples were digested for 4 h in 1 mL of 70% nitric acid at 85°C. Samples were cooled at room temperature, centrifuged at 5000 rpm for 1 min, diluted into 34 mL double-deionized water (2% nitric acid solution), vortexed, and assayed by ICP-MS.

### 2.5. Quantitative Determination of Lipid Peroxidation

Lipid peroxidation was determined by measuring hepatic malondialdehyde (MDA) content. We incubated 50 *μ*L protein from the tissues with 8.1% sodium dodecyl sulfate (SDS), 20% acetic acid, and 0.57% thiobarbituric acid at 90°C for 70 min. After cooling the samples on ice, 100 μL of double-distilled water was added to each tube, followed by 15 min of centrifugation at 4000 × g. The fluorescence intensity, reflecting the MDA content of each sample, was detected using a microplate reader (SpectraMax M3; Molecular Devices, Sunnyvale, CA, USA) under specific wavelength conditions (optical density, OD = 540 *μ*m). The final MDA content in each sample was calculated as follows: MDA = (OD of sample − OD of standard) × 178/protein concentration (mmol/mg).

### 2.6. Histological Analysis

Excised liver tissue specimens were fixed in 10% formalin and then treated in graded alcohol and xylene before being embedded in paraffin. The paraffin slices (5 millimeters) were deparaffinized and rehydrated before staining with hematoxylin and eosin (H&E) according to standard protocols. For immunohistochemical staining, endogenous peroxidases were blocked by treatment with 0.3% hydrogen peroxide in methanol for 30 min after deparaffinization and hydration. Antigen retrieval was performed using retrieval solution in a decloaking chamber (Biocare Medical, Concord, CA, USA) at 95°C for 25 min after three PBS washes and then cooled to room temperature. Nonspecific binding was blocked for 30 min with 5% bovine serum albumin in PBS. Sections were incubated with anti-alpha 1 fetoprotein antibody (AFP, 1 : 200 dilution; ab46799; Abcam) overnight at 4°C. After sections were washed thrice with PBS, they were incubated with horseradish peroxidase-conjugated secondary antibodies (1 : 500 dilution in PBS) for 1 h at room temperature. For color development, sections were treated with peroxidase substrate DAB (3,3-diaminobenzidine) in the developing system (Vector Laboratories, Burlingame, CA) and counterstained with hematoxylin. Lipid accumulation in liver tissues was analyzed using Oil Red O staining. Frozen liver tissue slices (10 *μ*m) were fixed in 10% formalin for 10 min before being rinsed in water. The slides were then submerged in 60% isopropanol and incubated for 18 min at room temperature in Oil Red O solution (saturated Oil Red O isopropanol solution diluted 4 : 6 in 60% isopropanol, Sigma-Aldrich, St. Louis, MO, USA). The slides were cleaned twice with 60% isopropanol and counterstained for 30 s with hematoxylin (DAKO, Carpinteria, CA, USA).

The stained sections were then viewed using an Olympus BX43 microscope (Olympus life science, Tokyo, Japan) and analyzed with ImageJ 1.44 software (Media Cybernetics, Bethesda, MD, USA). To investigate the lipid droplet sizes, we analyzed five fields of each mouse under the microscopy at 20 times magnification. The long diameters of 10 largest lipid droplets in each of the five fields were measured, and an average was calculated for each mouse.

### 2.7. Nuclear Protein Extraction

Nuclear proteins were extracted using a nuclear extraction kit (Cat#113474, Abcam, Cambridge, MA, USA) as follows: small pieces of tissue were weighed and cut. The tissue was homogenized with preextraction buffer containing dithiothreitol (DTT) solution and centrifuged, and the supernatant was removed. The nuclear sediment was mixed with the extraction buffer (DTT solution and a protease inhibitor cocktail), and the extract was vortexed on ice. After centrifugation of the suspension, the supernatant was collected.

### 2.8. Western Blot Analysis

For the western blot assay, liver tissues were collected and lysed. Lysate proteins from liver tissues were separated using 8%–12% SDS polyacrylamide gel electrophoresis and electrotransferred onto a nitrocellulose membrane. The protein blots were probed with antibodies against the cluster of differentiation 36 (CD36, 1 : 1000 dilution; ab133625; Abcam, Cambridge, MA, USA); peroxisome proliferator-activated receptor- (PPAR-) gamma co-activator-1 alpha (PGC1*α*, 1 : 1000 dilution; ab54481; Abcam, Cambridge, MA, USA); vascular cell adhesion molecule-1 (VCAM, 1 : 1000 dilution; ab134047; Abcam, Cambridge, MA, USA); NOD-, LRR-, and pyrin domain-containing protein 3 (NLRP3, 1 : 1000 dilution; ab210491; Abcam, Cambridge, MA, USA); interleukin-1*β* (IL-1*β*, 1 : 1000 dilution; ab9722; Abcam, Cambridge, MA, USA); PPAR*α* (1.0 *μ*g/mL dilution; PA1-822A, Invitrogen, Waltham, MA, USA); fatty acid-binding protein 1 (FABP1, 1 : 1000 dilution; 5352s; Cell Signaling Technology, Danvers, MA, USA); proliferating cell nuclear antigen (PCNA,1 : 1000 dilution; ab15497; Abcam, Cambridge, MA, USA); Histone3 (1 : 2000 dilution; 4499s; Cell Signaling Technology, Danvers, MA, USA); *α*-tubulin (1 : 1000 dilution; 2144s; Cell Signaling Technology, Danvers, MA, USA); nuclear factor-kappa B (NF-*κ*B, 1 : 1000 dilution; 8242s; Cell Signaling Technology, Danvers, MA, USA); phosphorylated NF-*κ*B (1 : 1000 dilution; 3033s; Cell Signaling Technology, Danvers, MA, USA); signal transducer and activator of transcription 3 (STAT3, 1 : 1000 dilution; 9139s; Cell Signaling Technology, Danvers, MA, USA); and phosphorylated STAT3 (1 : 1000 dilution; 9134s; Cell Signaling Technology, Danvers, MA, USA). The immunoreactive bands were detected using enhanced chemiluminescence reagents after incubation with appropriate secondary antibodies (Cell Signaling Technology, Danvers, MA, USA) conjugated with horseradish peroxidase (Bio-Rad, Hercules, CA, USA). The amount of proteins was analyzed using Image Lab analysis software (Bio-Rad, Hercules, CA) and normalized against their corresponding controls.

### 2.9. Statistical Analysis

Experimental data are presented as mean ± standard deviation (SD) (*n* = 3–7 per group). Statistical analyses were performed using one-way analysis of variance with the Tukey post hoc test using Prism 7.0 (GraphPad Software, San Diego, CA, USA). Statistical significance was defined as *p* < 0.05.

## 3. Results

### 3.1. Effects of Early-Life Exposure to Low-Dose Cd on Offspring General Health

To begin to elucidate the role of early-life, low-dose Cd exposure on adverse health effects in adulthood, we measured body weights starting at weaning (3 weeks of age) until 29 weeks of age in male (Figure 1(b)) and female (Figure 1(c)) offspring. For males, no significant differences in dynamic body weights were observed among the three groups of mice until 10 weeks of age; however, afterward, body weights significantly increased in the Con-Can mice (with DEN/HFCD) and further increased in the Cd-Can mice in a time-dependent manner compared to control mice. In females, before 12 weeks of age, no significant difference was observed in body weight among the three groups of mice; however, after 12 weeks, both Con-Can and Cd-Can mice showed a significant time-dependent increase in body weight, compared to controls, with Cd-Can mice gaining more weight compared to Con-Can mice.

At the termination of the experiments (offspring at 29 weeks old), fasting glucose levels in males were elevated in both Con-Can and Cd-Can mice (Figure 2(a)). The glucose tolerance test showed a significant increase in the area under the curves (AUC) for the Con-Can and Cd-Can mice, although the difference was not statistically significant (Figures 2(b) and 2(c)), suggesting the existence of a certain degree of insulin resistance in both groups. Similar effects of early-life exposure to low-dose Cd on fasting glucose levels and glucose tolerance were also observed in female mice (Figures 2(d)–2(f)), but the AUC value of the Cd-Can group was significantly higher than that of the Con-Can group (Figure 2(f)), suggesting that female offspring are more sensitive to HFCD diet-induced insulin resistance than male offspring.

Considering the similar results between male and female offspring, we focused on male offspring for the following experiments, otherwise specifically noticed. First, serum assays for male offspring showed no significant changes in triglyceride levels among the groups (Figure 2(g)), but there was a slight increase in cholesterol levels (Figure 2(h)) and ALT levels (Figure 2(i)) in Con-Can mice and a further increase in the Cd-Can mice.

### 3.2. Effects of Early-Life Exposure to Low-Dose Cd on Offspring's Liver Levels of Cd and Essential Metals (Zinc, Copper, and Iron)

Next, we examined whether early-life exposure to low-dose Cd affected liver metal levels in adulthood using ICP-MS. The first measurement of liver metals in the offspring was done at 3 weeks of age, before HCC induction. We found a significant increase in the liver Cd levels in the offspring with early-life exposure to Cd compared to the control (Figure 3(a)), confirming that early-life exposure to Cd via maternal and breastfeeding increased Cd accumulation in the offspring's liver. However, the mildly increased Cd accumulation did not affect the liver zinc, copper, or iron levels at weaning (3 weeks) (Figure 3(a)). The offspring's liver metals were also examined at 26 (Figure 3(b)) and 29 (Figure 3(c)) weeks of age. There was no significant Cd accumulation in the liver of offspring with early-life exposure to Cd at 26 and 29 weeks of age and no effect on the liver zinc level. However, both copper and iron levels were significantly lower in both the Con-Can and Cd-Can groups, suggesting that copper and iron deficiency at the late stage is most likely due to the effect of DEN/HFCD.

### 3.3. Early-Life Exposure to Low-Dose Cd Increases Offspring Susceptibility to DEN/HFCD Diet-Induced Liver Cancer

Based on a previous study that showed DEN/HFCD diet induced a high incidence of tumors after 20 weeks [20], we examined whether HCC was induced at the 23^rd^ week post-DEN/HFCD diet (i.e., 26 weeks old) by sacrificing three male and three female mice from each group. In male mice, no liver cancer was observed in controls, but cancer was detected in two of the three Con-Can mice and in all the three Cd-Can mice (Table 1). For each liver, there were four and five tumors on the liver surface in the two Con-Can mice but five or six tumors in the three Cd-Can mice (Figure 4(a)). Although there were only three mice in each group, a high incidence of liver tumor and more tumor nodules were observed in each liver of the Cd-Can mice compared to the Con-Can mice. These results suggest increased susceptibility of these mice to DEN/HFCD diet-induced liver cancer. However, only one female mouse in the Cd-Can group developed tumor (Table 1), with only one nodule on the liver surface (Figure 4(b)).

At 29 weeks of age, all the male mice in the Cd-Can and Con-Can groups had tumors (Table 1), while only half of the female mice in both the Con-Can and Cd-Can groups had tumors (Table 1), demonstrating a lower incidence of liver cancer in female mice.

Liver weight has been used as an indirect index of the severity of tumor burden, but we did not find a significant difference among the groups of female offspring (Figure 4(d)), and there was no significant difference in the tumor numbers between the females in Con-Can and Cd-Can groups (Figure 4(c)). However, we found an increasing trend in the liver weights of Con-Can mice and significantly increased liver weights in the Cd-Can mice compared to the Con-Can mice (Figure 4(e)).  Figure 4(f) shows the images of representative livers from the three groups, indicating more nodules in the Cd-Can group compared to the Con-Can group, which was confirmed by quantitative analysis of the nodule numbers per liver (Figure 4(g)). In addition, we observed larger tumor sizes (1.5–2 and 2.5–5 mm, Figure 4(h)) in the Cd-Can group than in the Con-Can group.

### 3.4. Cellular Features of Liver Cancer and Peritumor Analysis

To further define the features of liver cancer, H&E staining was performed for inflammatory cells and steatosis.  Figure 5(a) shows the tumor in the liver section, and the peritumor tissue displays severe steatosis, ballooned hepatocytes, and inflammatory cell infiltration.

Alpha-fetoprotein (AFP) is produced primarily by the liver in a developing fetus or as a result of liver damage and certain cancers. Immunohistochemical staining showed a significant increase in AFP-positive cells in the nodules of Cd-Can livers and Con-Can livers, but the former had a significantly higher increase than the latter (Figure 5(b)).

PCNA, a marker of proliferative nuclei, was stained to confirm the proliferation of the liver cells (Figure 5(c)). The number of cells positive for PCNA was significantly increased in the liver with the following features: (1) the control group had some scattered cells with weakly positive staining of the nucleus; (2) weak positive and scattered strong positive nuclear staining in the nontumor areas of the Con-Can and Cd-Can groups; and (3) strong positive nuclear staining localized in the tumor areas of the Con-Can and Cd-Can groups (Figure 5(c), Table 2). The upregulated PCNA expression was also confirmed by western blotting with protein lysis from liver nontumor and tumor areas (Figure 5(d)), although the difference was not statistically significant.

### 3.5. Increased Susceptibility of the Offspring to Liver Cancer in Cd-Can Mice by Early-Life Exposure to Low-Dose Cd Is Associated with Chronic Hepatic Inflammation and Lipid Metabolism Disturbance

HCC is known to be associated with chronic inflammation [21]. The Con-Can mice in this study showed higher body weight gain and insulin resistance (Figures 1 and 2), two important features of metabolic syndrome and risk factors for systemic and chronic inflammation; therefore, we examined the protein expression of NF-*κ*B, STAT3, VCAM, NLRP3, and IL-1*β* in peritumor tissues (Figure 6). The phosphorylation of NF-*κ*B and STAT3 increased in the cancer groups, especially in the Cd-Can group (Figures 6(a) and 6(b)). Similarly, cancer groups, particularly the Cd-Can group, displayed higher protein levels of VCAM, NLRP3, and IL-1*β*, as detected by western blotting (Figures 6(c)–6(e)).

Regarding the potential mechanisms underlying metabolic syndrome accompanied by chronic inflammation, we considered lipid metabolic disturbance, one of the main cellular features of metabolic syndrome that might be involved in the induction of chronic hepatic inflammation. Therefore, we tested fatty acid metabolism-related markers in the peritumor liver tissue. As a key fatty acid translocase, CD36 expression was elevated in mice subjected to HCC induction, especially in the Cd-Can group (Figure 7(a)). Western blotting also revealed a decreasing trend in the expression of FABP1, a member of intracellular fatty acid-binding and transporting proteins into the mitochondria for *β*-oxidation, in the Con-Can group compared to the control and in Cd-Can groups compared to the Con-Can group (Figure 7(b)).

Notably, the main mechanism for fatty acid disposal in the liver is *β*-oxidation in the mitochondria or storage as triglycerides. Accordingly, the protein levels of PPAR*α* and PGC1*α* were detected by western blotting and were significantly decreased in both cancer groups, particularly in the Cd-Can group (Figures 7(c) and 7(d)). Oil Red O staining demonstrated more lipid droplets in the liver tissue in the cancer groups than in the control group (Figures 8(a) and 8(b)) and larger lipid droplets in Cd-Con group than in the Con-Can group (Figure 8(c)). Similarly, the cancer groups showed higher liver tissue triglyceride levels compared with the control group, but the Cd-Can group showed a relatively lower increase compared with the Con-Can group (Figure 8(d)), which is consistent with the triglyceride levels in the blood (Figure 2(g)). Lipid peroxidation, an oxidative stress marker, was measured using the MDA assay, which showed an increase in the cancer groups. Of note, the Cd-Can group showed the highest level of MDA expression among the three groups (Figure 8(e)).

## 4. Discussion

In recent years, the hazardous nonessential metal Cd has been considered an endocrine disruptor [22], by the attributed association with obesity, diabetes, and carcinogenesis. In addition to Cd-induced acute or chronic target organ damage, early-life Cd exposure-related health risks have received more attention [23–25]. Jackson et al. showed that gestational Cd exposure induced preneoplastic lesions in the liver of female mice in early adulthood (about 3 months old) [19]. However, whether perinatal Cd exposure increases the susceptibility of the offspring to secondary stress-induced liver cancer remains unexplored. Our study indicates that early-life (prenatal to early postnatal) exposure to low-dose Cd increased DEN/HFCD diet-induced liver cancer in mice, which is associated with hepatic lipid metabolism disturbance and chronic inflammation.

In this study, we showed no body weight difference at weaning between offspring with and without early-life Cd exposure. No significant body weight difference was observed between HFCD diet-fed and normal diet-fed mice until 10 weeks of age for males and until 12 weeks of age for females. Afterward, the Con-Can mice showed a significant increase in body weight in a time-dependent manner, with the Cd-Can mice having a further increase. At 29 weeks of age, the body weight of Cd-Can male mice was 16.30% higher than that of the age-matched Con-Can group. In the female group, the increase was 40.15%. This finding is similar to that of a previous study showing that pre- and postnatal exposure to 0.5 ppm CdCl_2_ induced a delayed obesity in female CD-1 mouse offspring; however, this obesogenic effect of Cd in the previous study was not observed in male offspring [19]. The gender differences between our studies may be attributed to the mouse strain since we used C57BL/6J mice exposed to Cd in early life. Green et al. showed that in humans, the presence of Cd in maternal blood during pregnancy was associated with an increased risk of obesity in the offspring by five years of age with a steep growth [26]. However, data are lacking on the association between perinatal Cd exposure and body weight gain in adulthood in humans. The maternal Cd burden is associated with differential methylation of the fetal genome [15]. In Cowley et al.'s study, sequencing of the cord blood of newborns with maternal Cd exposure revealed that body mass index (BMI) is one of the top three functional gene categories with differentially methylated regions [27]. In our study, the HFCD diet induced an increase in fasting glucose levels in both males and females. Early-life exposure to low-dose Cd increased the fasting glucose levels in males compared with the same sex and diet controls. In females, the peak glucose concentration in response to glucose infusion increased in the HFCD-diet groups regardless of early-life Cd exposure. However, early-life exposure to low-dose Cd reduced the rate of glucose clearance, in line with two previous studies [18, 19].

The metal measurement in this study showed that at the time of weaning, the Cd level in the liver was higher in the mice with early-life Cd exposure compared with the control mice, but this difference disappeared at 26 and 29 weeks of age. This result is similar to that of a previous study, which showed higher liver Cd levels in Wistar rats with early-life Cd exposure at weaning than in the age-matched controls [18]. Two months after birth, the liver Cd level of rats with low-dose early-life Cd exposure was similar to that of age-matched control rats, and in the group exposed to Cd concentrations equivalent to our study, the liver Cd level of rats also decreased compared to that at weaning. We also tested for the zinc, iron, and copper levels in the liver at the time points mentioned above. The concentrations of these essential metals did not differ between the groups with and without Cd exposure at weaning, indicating that the increased Cd does not directly affect these essential metal levels at weaning. However, apart from zinc, iron and copper concentrations significantly decreased in the cancer groups at 26 and 29 weeks of age, which may contribute to essential metal dyshomeostasis in the liver and eventually contribute to liver cancer development.

In this study, we showed that at 26 weeks of age, all the three mice from the male Cd-Can group developed an average of five tumors on the liver surface. However, in the Con-Can group, two out of three mice developed tumors with an average of four tumors per mouse on the liver surface. At 29 weeks of age, all male mice in the Con-Can and Cd-Can groups had developed liver tumors. Quantitative analysis showed more tumors per liver and larger tumor sizes in the Cd-Can group compared to the Con-Can group. The differences between the Con-Can and Cd-Can groups suggest that early-life low-dose Cd exposure increases the susceptibility to liver tumor induction by the DEN/HFCD diet. In contrast, only one female in the Cd-Can group developed liver tumors at 26 weeks of age. At 29 weeks of age, three out of six mice developed liver tumors in both Con-Can and Cd-Can female mice. The gender difference in the liver tumor incidence is comparable to that observed in a previous study [28] that found that estrogen is a protective factor for liver cancer. Considering the comparable liver Cd levels of mice with or without early-life low Cd exposure at 26 and 29 weeks of age and a higher body weight gain in the Cd-Can mice, we hypothesize that the early-life low Cd exposure may accelerate liver tumor development, probably by impairing energy metabolism and consequent obesity.

A clear relationship between obesity and liver tumors is well established. Obesity is a major risk factor for metabolic syndrome, steatosis, and steatohepatitis, which can lead to HCC [29, 30]. The HFCD diet used in this study has been used previously in mice to induce steatohepatitis [30, 31]. In our study, early-life low Cd exposure led to greater body weight gain. In the peritumor liver tissue, fatty acid metabolism was disrupted by the DEN/HFCD diet, which was accelerated by early-life low Cd exposure. CD36, a fatty acid translocase, increases free fatty acid uptake [32]. In the Con-Can and Cd-Can groups, liver tissue showed high CD36 expression, especially in Cd-Can mice, which resulted in higher intracellular fatty acid concentrations. FABP1 is the intracellular conduit for fatty acid delivery to enzymes [33]. However, FABP1 expression in our study lacked a comparable increase in the Con-Can and Cd-Can groups, despite the higher CD36 expression. In addition, the low FABP1 expression in the Cd-Can group leads to insufficient transfer of fatty acids into mitochondria for *β*-oxidation, which is a major disposal mechanism of fatty acids. Furthermore, the present study showed a reduction in PPAR*α* and PGC-1*α* expression in Con-Can and Cd-Can groups, with a greater decrease in the latter, suggesting impaired *β*-oxidation in the mitochondria. These findings are comparable to those of a recent study, which showed a marked decrease in the hepatic expression of PGC-1*α* and its target genes involved in gluconeogenesis in a mouse model of HCC induced by a choline-deficient diet and in primary human HCC [34]. These findings show that hepatic mitochondrial dysfunction or maladaptation contributes to the detrimental effects on hepatocyte bioenergetics, reactive oxygen species homeostasis, endoplasmic reticulum response, inflammation, and cell death, leading to nonalcoholic steatohepatitis (NASH) and HCC [35].

Regarding lipotoxicity and oxidative stress, we stained the liver with Oil Red O and showed a significant increase in the lipid droplets in the Con-Can and Cd-Can groups without significant differences between the two groups. However, MDA, an index of lipid peroxidation or oxidative stress, significantly increased in both Con-Can and Cd-Can groups but was significantly higher in the latter than in the former. However, the liver triglyceride level was lower in the Cd-Can group than in the Con-Can group. The downregulated formation of esterified triglyceride combined with decreased mitochondrial *β*-oxidation in the Cd-Can group compared with the Con-Can group indicates impaired fatty acid disposal. Notably, the increased fatty acid uptake and decreased fatty acid disposal indicate a greater fatty acid burden in the peritumor liver tissue, which contributes to worse lipotoxicity (Figure 8).

The enhanced lipotoxicity in the Cd-Can group is one of the major mechanisms that induce inflammation in the NASH model [36]. In our study, the mice in the Cd-Can group displayed higher lipotoxicity, accompanied by higher levels of inflammation-related markers. The elevated phosphorylation of NF-*κ*B in our study is consistent with the findings of Wolf et al., who showed that canonical NF-*κ*B signaling mediated the NASH-to-HCC transition in the HFCD-fed mouse NASH model [30].

Perinatal Cd exposure as an endocrine disruptor has been explored in Jackson et al.'s study, and it also contributed to liver preneoplastic lesions in early adulthood [19]. However, whether perinatal Cd exposure increases the susceptibility of offspring to liver cancer or not remains unknown. In this study, we investigated whether early-life low Cd exposure accelerates HFCD diet combined with DEN-induced liver tumors. We have shown that early-life low Cd exposure leads to a higher body weight gain in both male and female mice. For females, early-life low Cd exposure worsens insulin intolerance, but there is no evidence that it enhanced the HFCD diet combined with DEN-induced liver tumor. In contrast, early-life low Cd exposure induces more and larger liver tumors with earlier onset, which may be attributed to impaired energy metabolism, increased fatty acid-induced lipotoxicity, and subsequent chronic inflammation.

This study has potential limitation. It revealed that early-life Cd exposure increases susceptibility to liver tumors in mice, possibly by interfering with fatty acid metabolism. The reason behind this, however, is unknown. We and others have shown that Cd exposure causes epigenetic alterations [14] that also affects the offspring [27]. The epigenetic alterations of the functional gene categories, especially the metabolism-related genes will be estimated at weaning in the future study.

## Figures and Tables

**Figure 1:** Animal model for this study (a). The dynamic body weights of male (b) and female (c) offspring were recorded and expressed as mean (*n* = 6-10). ^∗∗^*p* < 0.01 and ^∗∗∗∗^*p* < 0.0001, Con-Can vs. control; ^##^*p* < 0.01 and ^###^*p* < 0.001, Cd-Can vs. Con-Can.

**Figure 2:** Metabolic alteration. The fasting blood glucose of male (a) and female (d) mice, the IPGTT results of male (b) and female (e) mice, and the quantitative analysis results of male (c) and female mice (f). Blood triglyceride (g), cholesterol (h), and ALT (i) levels in male mice. Quantitative data are expressed as the mean ± SEM (*n* = 6-7). ^∗^*p* < 0.05, ^∗∗^*p* < 0.01, and ^∗∗∗^*p* < 0.001, Con-Can vs. control; ^#^*p* < 0.05, Cd-Can vs. Con-Can. ALT: alanine aminotransferase; IPGTT: intraperitoneal glucose tolerance test; SEM: standard error of the mean.

**Figure 3:** Cd, zinc, copper, and iron levels of the liver. Cd, zinc, copper, and iron levels in the liver at weaning (a), 26 weeks of age (b), and 29 weeks of age (c) were determined by ICP-MS. Quantitative data are expressed as mean ± SEM (*n* = 3-10). ^∗∗^*p* < 0.01, Cd vs. control; ^∗∗∗∗^*p* < 0.0001, Con-Can vs. control. Cd: cadmium; ICP-MS: inductively coupled plasma mass spectrometry; SEM: standard error of the mean.

**Figure 4:** Tumor data of 26- and 29-week-old male and female mice. The number of tumors on the liver surface of male mice at 26 weeks of age (a) and 29 weeks of age (g) and female mice at 26 (b) and 29 (c) weeks of age was recorded. The ratio of liver weight to tibia length in female (d) and male (e) mice. Macroscopy of 29-week-old male mouse liver (f), with the arrowhead pointing towards HCC. The size of liver surface tumors for male mice in the Con-Can and Cd-Con groups (h). Quantitative data are expressed as the mean ± SEM, *n* = 3-7. ^#^*p* < 0.05, Cd-Can vs. Con-Can. HCC: hepatocellular carcinoma; SEM: standard error of the mean.

**Figure 5:** Biological characteristics of the liver tumor. Representative images of hematoxylin and eosin- (H&E-) stained (a), AFP (b), and PCNA- (c) stained liver sections. The AFP IHC staining-positive area (%) is labeled as the mean ± SEM. PCNA protein expression was detected in the nucleus of tumor and nontumor liver tissue from male mice, and Histone3 was used as a loading control for western blot assay (d). Quantitative data were normalized to the control and expressed as the mean ± SEM. Scale bar represents 200 *μ*m. AFP: alpha fetoprotein; IHC: immunohistochemical staining; PCNA: proliferating cell nuclear antigen; SEM: standard error of the mean.

**Figure 6:** Inflammation-related protein expression in the peritumor liver tissue. Protein expression of phosphorylation and total NF-*κ*B (a), phosphorylation and total STAT3 (b), VCAM (c), NLRP3 (d), and IL-1*β* (e) in male mouse peritumor liver tissue was detected, and *α*-tubulin was used as the loading control for western blot assay. Quantitative data were normalized to the control and expressed as mean ± SEM (*n* = 7). ^∗^*p* < 0.05 and ^∗∗^*p* < 0.01, Con-Can vs. control; ^#^*p* < 0.05 and ^##^*p* < 0.01, Cd-Can vs. Con-Can. NF-*κ*B: nuclear factor-kappa B; STAT3: signal transducer and activator of transcription 3; VCAM: vascular cell adhesion molecule-1; NLRP3: NOD-, LRR-, and pyrin domain-containing protein 3; IL-1*β*: interleukin-1*β*; SEM: standard error of the mean.

**Figure 7:** Fatty acid metabolism-related protein expression in the peritumor liver tissue. Protein expression of CD36 (a), FABP1 (b), PPAR*α* (c), and PGC1*α* (d) in the peritumor liver tissue of male mice was detected, and *α*-tubulin was used as a loading control for western blot assay. Quantitative data were normalized to the control and expressed as mean ± SEM (*n* = 7). ^∗^*p* < 0.05 and ^∗∗∗^*p* < 0.01, Con-Can vs. control; ^#^*p* < 0.05, Cd-Can vs. Con-Can. CD36: cluster of differentiation 36; FABP1: fatty acid-binding protein 1; PPAR*α*: peroxisome proliferator-activated receptor alpha; PGC1*α*: peroxisome co-activator-1 alpha; SEM: standard error of the mean.

**Figure 8:** Hepatic lipid accumulation and potential mechanistic illustration. Oil Red O staining of the peritumor liver tissue (a) and the positive area quantitative analysis (b). Panel (c) shows the difference in lipid droplet sizes between Con-Can and Cd-Can groups. The triglyceride (d) and malondialdehyde levels (e) of the peritumor liver tissue in each group were evaluated. Quantitative data are expressed as mean ± SEM, *n* = 6-7. Panel (f) is the illustration of free fatty acid metabolism alteration of peritumor liver tissue. Increased CD36 expression mediates the free fatty acid uptake in Con-Can and Cd-Can groups, especially in the Cd-Can groups. The *β*-oxidation in mitochondria and formation of esterified triglyceride are the major disposal mechanism of fatty acid, and these were decreased in the Cd-Can group compared with the Con-Can group. Increased uptake and decreased disposal result in the increase of hepatocyte free fatty acid flux, which mediated the lipotoxicity, followed by carcinogen; red arrow, Cd-Can vs. Con-Can. The scale bar represents 100 *μ*m. ^∗^*p* < 0.05, ^∗∗^*p* < 0.01, and ^∗∗∗∗^*p* < 0.0001, Con-Can vs. control; ^#^*p* < 0.05 and ^##^*p* < 0.01, Cd-Can vs. Con-Can. CD36: cluster of differentiation 36; SEM: standard error of the mean.

**Table 1:** Incidence of liver tumor.

		Control (*n*/*n*)	Con-Can (*n*/*n*)	Cd-Can (*n*/*n*)
26 weeks old	Male	0/3	2/3	3/3
	Female	0/3	0/3	1/3
29 weeks old	Male	0/6	7/7	7/7
	Female	0/6	3/6	3/6

**Table 2:** Half-quantitative data of PCNA IHC staining.

		Non-T	T1	T2	T3	T4	T5	T6	T7	T8
Con-Can	No. 1	++	+++							
	No. 2	++	+++	++	++	++				
	No. 3	+	++	++	+++	++	+++	++	+++	+++
	No. 4	+++								
	No. 5	+	+	+	++	++	++			
	No. 6	−~+	−~+	+						
	No. 7	−	−~+	+						
Cd-Can	No. 1	−~+	−~+	+	+	+	+	+	++	
	No. 2	−~+	++	++	++	++	+	+	+	+
	No. 3	−~+	+	++	++	+++				
	No. 4	−~+	+	+						
	No. 5	−~+	+	+	++					
	No. 6	−~+	−~+	+	++					
	No. 7	−~+	−~+	−~+	−~+	+	+	+	+	++

Legends: Non-T: nontumor zone; T: tumor zone. −: negative. +: 0-5 strong positive-stained nuclei in every 10x field of view of Non-T or in one-fourth 10x field of view of T. ++: 6-10 strong positive-stained nuclei in every 10x field of view of Non-T or in one-fourth 10x field of view of T. +++: >10 strong positive-stained nuclei in every 10x field of view of Non-T or in one-fourth 10x field of view of T.

## Data Availability

The data used to support the findings of this study are included within the article.
